# Kinematic Calibration of a Parallel 2-UPS/RRR Ankle Rehabilitation Robot

**DOI:** 10.1155/2020/3053629

**Published:** 2020-09-03

**Authors:** Mingjie Dong, Yuan Kong, Jianfeng Li, Wenpei Fan

**Affiliations:** Beijing Key Laboratory of Advanced Manufacturing Technology, Faculty of Materials and Manufacturing, Beijing University of Technology, No. 100 Pingleiyuan, Chaoyang District, Beijing, China

## Abstract

In order to better perform rehabilitation training on the ankle joint complex in the direction of dorsiflexion/plantarflexion and inversion/eversion, especially when performing the isokinetic muscle strength exercise, we need to calibrate the kinematic model to improve its control precision. The ankle rehabilitation robot we develop is a parallel mechanism, with its movements in the two directions driven by two linear motors. Inverse solution of positions is deduced and the output lengths of the two UPS kinematic branches are calibrated in the directions of dorsiflexion, plantarflexion, inversion, and eversion, respectively. Motion of each branch in different directions is fitted in high-order form according to experimental data. Variances, standard deviation, and goodness of fit are taken into consideration when choosing the best fitting curve, which ensures that each calibration can match the most appropriate fitting curve. Experiments are conducted to verify the effectiveness of the kinematic calibration after finishing the calibration, and the errors before and after calibration of the two kinematic chains in different directions are compared, respectively, which shows that the accuracy after calibration has been significantly improved.

## 1. Introduction

Rehabilitation training is an effective way to help patients restore their ankle joint complex's (AJC) motor abilities for patients with ankle injuries. The movement of AJC has three Degrees of Freedom (DOFs), Dorsiflexion/Plantarflexion (DO/PL), Inversion/Eversion (IN/EV), and Adduction/Abduction (AD/AB) [1], with its coordinate system definition shown as in Figure 1.

To augment conventional physical therapy, many robotic ankle rehabilitation devices have been developed to provide repetitive, task-specific, interactive treatment of the impaired limb and monitor its motor recovery [2–6]. Passive rehabilitation training, which means that the AJC is driven by the robot for rehabilitation at a predetermined trajectory, is often used in the early stage of ankle therapy. Many ankle rehabilitation robots have realized the trajectory tracking control for passive rehabilitation training [7–9]. To improve the effect of rehabilitation training, many active rehabilitation training methods including the active participation of patients have been developed such as the ARBOT [5], CARR [10], and Anklebot [11]. Among different kinds of ankle rehabilitation robots, the platform ones are better suited for ankle exercises [12], and parallel mechanism is the most common among them with the above-mentioned exercise modes [5, 6, 13, 14].

Besides that, isometric and isotonic exercises have also been developed for muscle strength exercises of AJC [5, 15]. However, there was no isokinetic muscle strength exercise specially developed for ankle rehabilitation robot, during which the exercise speed is constant, while the resistance encountered varies with the degree of exertion, so that the muscle tension of the moving ankle maintains the optimal state of strength training [16], and the isokinetic muscle strength exercise is usually used for strength training with only one DOF per time. There have been isokinetic exercises used for joint rehabilitation, such as the IsoMed-2000 developed by D. & R. Ferstl, Germany [17].

To realize the isokinetic muscle strength exercise in DO/PL and IN/EV direction using our developed 2-UPS/RRR parallel ankle rehabilitation robot (PARR), we need to have the precise kinematic model of the two UPS kinematic branches. U, P, S, and R stand for universal, prismatic, spherical, and revolute joint, respectively, and the underlined letter represents the actuated joint. Considering machining and assembly errors, the designed robot needs to be calibrated firstly to make the positional inverse solution obtained by theoretical analysis more accurately.

The conventional approach toward kinematic calibration generally begins with formulating the problem in terms of constraint equations that are derived from the kinematic model of the robot. In the data acquisition phase, the pose of the moving platform and the corresponding actuated joint coordinates are obtained. Finally, a suitable optimization method utilizes the obtained data to determine the actual geometry [18]. In contrast, an alternative response surface methodology based method is proposed for performing kinematic calibration that does not require constraint equations and additional input data [19] and physical experiments have been conducted on a 3-PSS/S mechanism to evaluate the accuracy. By analyzing different objective functions for the parameter identification of parallel mechanisms and studying the influence in the position and orientation errors to improve their accuracy, a new objective function considering deviation terms is presented in [20], showing better kinematic parameters identification performance corresponding with passive joints that cannot be measured. Reference [21] proposes a stepwise approach to kinematic calibration of a 5-DOF Gantry-Tau parallel kinematic machine and achieves accuracy of about 20 micrometers for the base actuators by using measurements from a laser tracker and least-squares estimates of polynomial functions. Besides that, the kinematic calibration problem of overconstrained PM is addressed in [22] to improve accuracy and promote its practical application. Instead of establishing conventional error mapping model, a nonlinear error model is built by inserting geometric errors of parts to the real inverse position analysis, and the nonlinear identification equations are directly solved by optimization technique, with results showing very good orientation accuracy. Besides that, maximum likelihood estimation (MLE) is also often used for the calibration of robot or sensors [23].

In this work, we focus on the kinematic calibration of our 2-UPS/RRR PARR according to field experiments and high-order data fitting, with variances, standard deviation, and goodness of fit as the criterion of fitting evaluation. The rest of the paper is organized as follows.  Section 2 demonstrates the inverse solution of positions of the PARR. The kinematic calibration process is presented in Section 3.  Section 4 displays the experiments and validation, while conclusions are drawn and discussed in Section 5.

## 2. Inverse Solution of Positions of the PARR

### 2.1. Mechanical Design of the PARR

The mechanical structure of the developed 2-UPS/RRR PARR is shown in Figure 2. The mechanism is very simple with only a fixed base, a moving platform, two UPS kinematic branches, and a series RRR constraint branch, with its three rotation axes orthogonal to one point. It has three DOFs, with its three rotational DOFs, respectively, equipped with absolute encoders (CALT HAN28E5V360A2, analog output, resolution ±0.1%). The controller and the data acquisition system used in the robot are based on STM32F103ZET6, and the drivers used for the motors are HDT Servodrives DX060. The advantage of the designed PARR is that different patients' rotation centers of the AJC can coincide with the mechanism's rotation center in addition to its compact configuration. The estimated range of motion (ROM) of the human AJC in each direction is given in Table 1 [24], which is used as a reference to design the allowable motion range of the mechanical limits. Specifically, the limits for the rotation angles of the PARR are set as in Table 1, which determine the maximum allowable workspace (MAW) of the parallel mechanism and ensure that the robot is suitable for the left and right AJCs.

Details of mechanical design of the developed PARR are shown in our previous work [25]. During the ankle isokinetic muscle strength exercise, only the movements of DO/PL and IN/EV are usually considered. Therefore, here we just study the kinematic calibration of the two UPS kinematic branches actuated by two linear motors (SKF CAHB-10, driving distance of 150 mm).

### 2.2. Coordinate System of the Parallel Mechanism

The kinematic coordinate system of the parallel 2-UPS/RRR rehabilitation robot is shown as in Figure 3(a) [26]. The fixed coordinate system *O* − *X*_*o*_*Y*_*o*_*Z*_*o*_ and the moving coordinate system *M* − *X*_*m*_*Y*_*m*_*Z*_*m*_ are established at the rotation center of the mechanism coinciding at the initial position, all along the directions of three rotation axes. The moving coordinate system is fixed on the moving platform of the parallel mechanism. *A*_*i*_, *B*_*i*_, and *C*_*i*_(*i*=1,2,3) are the moving distances of the universal joint, spherical joint, and prismatic joint, respectively. The revolute joints *R*_1_, *R*_2_, and *R*_3_ are orthogonal to point “*O*,” with their rotation angles being *γ*, *α*, and *β* in turn, respectively, where *α* represents the angle of DO/PL and *β* represents the angle of IN/EV (right foot here), while *γ* denotes the angle of AD/AB, and the angle value is defined to be positive with counterclockwise rotation.

The coordinate system of the UPS branch is shown in Figure 3(b), where *A*_*i*_ − *X*_*A*,*i*_*Y*_*A*,*i*_*Z*_*A*,*i*_ is the coordinate system whose origin *A*_*i*_ is at the center of the universal joint with its axis **X**_*A*,*i*_ coinciding with the first axis of the universal joint and axis **Y**_*A*,*i*_ coinciding with second axis of the universal joint when the mechanism is in the initial position: **Z**_*A*,*i*_=**X**_*A*,*i*_ × **Y**_*A*,*i*_. *C*_*i*_ − *X*_*C*,*i*_*Y*_*C*,*i*_*Z*_*C*,*i*_ is the coordinate system whose origin *C*_*i*_ is at the center of the universal joint with its axis *Y*_*C*,*i*_ coinciding with the second axis of the universal joint and *Z*_*C*,*i*_ coinciding with the mechanism rod vector $\overset{⟶}{C_{i}D_{i}}$, while the axis **X**_*C*,*i*_=**Y**_*C*,*i*_ × **Z**_*C*,*i*_. *B*_*i*_ − *X*_*B*,*i*_*Y*_*B*,*i*_*Z*_*B*,*i*_ is the coordinate system whose origin *B*_*i*_ is at the center of the spherical joint with its three axes parallel with the corresponding axes of *C*_*i*_ − *X*_*C*,*i*_*Y*_*C*,*i*_*Z*_*C*,*i*_.

### 2.3. Inverse Solution of Positions

The inverse solution of positions is to deduce the inputs of three branches based on the output angles of the moving platform around the fixed coordinate system, that is, the above-mentioned *α*, *β*, and *γ*. The rotating matrix **R**_OM_ of the moving platform relative to the fixed base can be expressed as in the following equation:

(1) $$\begin{array}{c} R_{\text{OM}}=R\left(\gamma \right)R\left(\beta \right)R\left(\alpha \right)=\left[\begin{array}{ccc} c\gamma c\beta & -s\gamma c\alpha +c\gamma s\beta s\alpha & s\gamma s\alpha +c\gamma s\beta c\alpha \\ s\gamma c\beta & c\gamma c\alpha +s\gamma s\beta s\alpha & -c\gamma s\alpha +s\gamma s\beta c\alpha \\ -s\beta & c\beta s\alpha & c\beta c\alpha \end{array}\right], \end{array}$$

where *c* and *s* are the abbreviations of *cos* and *sin*, respectively. Then, the position vector of the center of spherical joint *B*_*i*_ in the *O* − *X*_*o*_*Y*_*o*_*Z*_*o*_ coordinate system can be expressed as in the following two equations, respectively:

(2) Bio=rM+ROMrMBi,

(3) Bio=liZC,i+rAi,

where **r**_*M*_ indicates the vector coordinates of point *M* in the *O* − *X*_*o*_*Y*_*o*_*Z*_*o*_ coordinate system, **r**_MB_*i*__ indicates the vector coordinates of point *B*_*i*_ in the *M* − *X*_*m*_*Y*_*m*_*Z*_*m*_ coordinate system and it is a constant, *l*_*i*_ indicates the total length of the *ith* UPS kinematic branches, and **r**_*A*_*i*__ indicates the vector coordinates of the point *A*_*i*_ in the *O* − *X*_*o*_*Y*_*o*_*Z*_*o*_ coordinate system and it is also a constant.

By combining (2) and (3), we can obtain (4), where || represents the length of the inside vector.

(4) $$\begin{array}{c} l_{i}=\left|r_{M}+R_{\text{OM}}r_{{\text{MB}}_{i}}-r_{A_{i}}\right|. \end{array}$$

According to the parameters of the developed 2-UPS/RRR PARR, the coordinate values of points *B*_1_ and *B*_2_ in the *M* − *X*_*m*_*Y*_*m*_*Z*_*m*_ coordinate system are (120,110, −4.5) and (−120,110, −4.5), respectively. The coordinate values of points *A*_1_ and *A*_2_ in the *O* − *X*_*o*_*Y*_*o*_*Z*_*o*_ coordinate system are (175,80, −406) and (−175,80, −406), respectively. Therefore, we can get the theoretical inverse solution of positions as in the following equation:

(5) $$\begin{array}{c} \left\{\begin{array}{c} l_{1}=\left|R_{\text{OM}}\left[\begin{array}{c} 120\\ 110\\ -4.5 \end{array}\right]-\left[\begin{array}{c} 175\\ 80\\ -406 \end{array}\right]\right|,\\ l_{2}=\left|R_{\text{OM}}\left[\begin{array}{c} -120\\ 110\\ -4.5 \end{array}\right]-\left[\begin{array}{c} -175\\ 80\\ -406 \end{array}\right]\right|. \end{array}\right. \end{array}$$

For our PARR, the angle of AD/AB *γ* is equal to the rotation angle of the servo motor due to the mechanical design of the parallel mechanism. Considering the isokinetic muscle strength exercise, the kinematic calibration here is mainly for the movement of DO/PL and IN/EV; that is, we need to compensate the output length of the two UPS kinematic branches to get the accurate relationship between *l*_*i*_ and *α* and *β*.

From (5), we can get the initial values of *l*_1_ and *l*_2_ as in the following equation:

(6) $$\begin{array}{c} l_{1}^{0}=l_{2}^{0}=\left|{\left[\begin{array}{c} -5530401.5 \end{array}\right]}^{T}\right|=406.3585. \end{array}$$

#### 2.3.1. Movement of DO/PL

During the movement of DO/PL (*β*=*γ*=0), we can deduce the values of *l*_1_ and *l*_2_ as follows:

(7) $$\begin{array}{c} \left\{\begin{array}{c} l_{1}=\left|\left[\begin{array}{ccc} 1 & 0 & 0\\ 0 & c\alpha & -s\alpha \\ 0 & s\alpha & c\alpha \end{array}\right]\left[\begin{array}{c} 120\\ 110\\ -4.5 \end{array}\right]-\left[\begin{array}{c} 175\\ 80\\ -406 \end{array}\right]\right|=\left|\left[\begin{array}{c} -55\\ 110c\alpha +4.5s\alpha -80\\ 110s\alpha -4.5c\alpha +406 \end{array}\right]\right|,\\ l_{2}=\left|\left[\begin{array}{ccc} 1 & 0 & 0\\ 0 & c\alpha & -s\alpha \\ 0 & s\alpha & c\alpha \end{array}\right]\left[\begin{array}{c} -120\\ 110\\ -4.5 \end{array}\right]-\left[\begin{array}{c} -175\\ 80\\ -406 \end{array}\right]\right|=\left|\left[\begin{array}{c} 55\\ 110c\alpha +4.5s\alpha -80\\ 110s\alpha -4.5c\alpha +406 \end{array}\right]\right|. \end{array}\right. \end{array}$$

The length changes of *l*_1_ and *l*_2_ during DO/PL are as in (8), from which we can see that Δ*l*_1_=Δ*l*_2_, and their direction is consistent.

(8) $$\begin{array}{c} \left\{\begin{array}{c} \Delta l_{1}=l_{1}-l_{1}^{0}=\left|\begin{array}{c} -55\\ 110c\alpha +4.5s\alpha -80\\ 110s\alpha -4.5c\alpha +406 \end{array}\right|-406.3585\text{,}\\ \Delta l_{2}=l_{2}-l_{2}^{0}=\left|\begin{array}{c} 55\\ 110c\alpha +4.5s\alpha -80\\ 110s\alpha -4.5c\alpha +406 \end{array}\right|-406.3585\text{.} \end{array}\right. \end{array}$$

#### 2.3.2. Movement of IN/EV

During the movement of IN/EV (*α*=*γ*=0), we can deduce the values of *l*_1_ and *l*_2_ as follows:

(9) $$\begin{array}{c} \left\{\begin{array}{c} l_{1}=\left|\left[\begin{array}{ccc} c\beta & 0 & s\beta \\ 0 & 1 & 0\\ -s\beta & 0 & c\beta \end{array}\right]\left[\begin{array}{c} 120\\ 110\\ -4.5 \end{array}\right]-\left[\begin{array}{c} 175\\ 80\\ -406 \end{array}\right]\right|=\left|\left[\begin{array}{c} 120c\beta -4.5s\beta -175\\ 30\\ -120s\beta -4.5c\beta +406 \end{array}\right]\right|,\\ l_{2}=\left|\left[\begin{array}{ccc} c\beta & 0 & s\beta \\ 0 & 1 & 0\\ -s\beta & 0 & c\beta \end{array}\right]\left[\begin{array}{c} -120\\ 110\\ -4.5 \end{array}\right]-\left[\begin{array}{c} -175\\ 80\\ -406 \end{array}\right]\right|=\left|\left[\begin{array}{c} -120c\beta -4.5s\beta +175\\ 30\\ 120s\beta -4.5c\beta +406 \end{array}\right]\right|. \end{array}\right. \end{array}$$

The length changes of *l*_1_ and *l*_2_ during IN/EV are as in the following equation:

(10) $$\begin{array}{c} \left\{\begin{array}{c} \Delta l_{1}=l_{1}-l_{1}^{0}=\left|\begin{array}{c} 120c\beta -4.5s\beta -175\\ 30\\ -120s\beta -4.5c\beta +406 \end{array}\right|-406.3585,\\ \Delta l_{2}=l_{2}-l_{2}^{0}=\left|\begin{array}{c} -120c\beta -4.5s\beta +175\\ 30\\ 120s\beta -4.5c\beta +406 \end{array}\right|-406.3585. \end{array}\right. \end{array}$$

We can see that Δ*l*_1_ ≠ Δ*l*_2_ during the movement of IN/EV when *β* ≠ 0 and they change in the opposite direction. Based on the above analysis, Δ*l*_1_ and Δ*l*_2_ can be calibrated simultaneously during DO/PL, while during IN/EV, Δ*l*_1_ and Δ*l*_2_ need to be calibrated separately.

## 3. Calibration Process of the Designed Parallel Mechanism

The error model of the kinematic calibration is as in (11), and we do not know the exact form of the errors in advance.

(11) $$\begin{array}{c} l_{i}=\left|r_{M}+R_{\text{OM}}r_{{\text{MB}}_{i}}-r_{A_{i}}\right|+\Delta l_{i}. \end{array}$$

During the calibration, firstly, we control the output lengths of *l*_1_ and *l*_2_ using the position controller for the two linear actuators to realize the movement of DO/PL and IN/EV, respectively. Secondly, we record the corresponding output angles of DO/PL and IN/EV, that is *α*, *β*, respectively. Finally, the recorded *α* and *β* are used to deduce the theoretical values of the lengths of *l*_1_ and *l*_2_ according to the inverse solution of positions. The difference between the theoretical values of *l*_1_ and *l*_2_ and the controlled lengths of *l*_1_ and *l*_2_ is used to calculate and compensate the errors.

### 3.1. Calibration of *l*_1_ and *l*_2_ in DO/PL Direction

The result of calibration in DO/PL is as in Figure 4, from which we can see that the error trends in DO and PL are different, so we calibrate them separately.

#### 3.1.1. Error Calibration of *l*_1_ and *l*_2_ in DO Direction

The second-order fitting, third-order fitting, fourth-order fitting, fifth-order fitting, and sixth-order fitting are, respectively, performed on the errors between actual and theoretical values of *l*_1_ and *l*_2_ during the movement of DO, with their fitting results shown as in Figure 5. In order to better analyze the results, we calculate the variances, standard deviations, and goodness of fit of each of the fitting values with the errors, as shown in Table 2, where Var, Std, and *R*^2^ represent the variance, standard deviation, and goodness of fit, respectively.

After comprehensive consideration of variances, standard deviations, goodness of fit, and computation complexity according to the fitting result, we define the criterion of choosing the optimal fitting curve as in the following equation:

(12) $$\begin{array}{c} \left\{\begin{array}{c} \text{Var}\leq 0.04\\ \text{Std}\leq 0.2\\ R^{2}\geq 0.6 \end{array}\right.. \end{array}$$

According to Figure 5 and Table 2, we choose fifth-order fitting as the optimal fitting curve of error compensation of *l*_1_ and *l*_2_ in DO direction as in the following equation:

(13) $$\begin{array}{c} \Delta l_{1}=\Delta l_{2}=1.4469\times 10^{-4}\alpha^{5}-0.0056\alpha^{4}+0.0781\alpha^{3}-0.4739\alpha^{2}+1.2322\alpha -0.136. \end{array}$$

#### 3.1.2. Error Calibration of *l*_1_ and *l*_2_ in PL Direction

The second-order fitting, third-order fitting, fourth-order fitting, fifth-order fitting, and sixth-order fitting are, respectively, performed on the errors between actual values and theoretical values of *l*_1_ and *l*_2_ during the movement of PL, with their fitting results as in Figure 6. The variance, standard deviation, and goodness of fit of each of the fitting values with the errors are shown in Table 3.

According to Figure 6 and Table 3, we choose second-order fitting as the optimal fitting curve of error compensation of *l*_1_ and *l*_2_ in PL direction as in the following equation:

(14) $$\begin{array}{c} \Delta l_{1}=\Delta l_{2}=-0.0035\alpha^{2}+0.0106\alpha -1.1415. \end{array}$$

### 3.2. Calibration of *l*_1_ in IN/EV Direction

The result of *l*_1_ calibration in the direction of IN/EV is as in Figure 7, from which we can see that the error trends in IN/EV are also different, so we will calibrate them separately.

#### 3.2.1. Error Calibration of *l*_1_ in IN Direction

The second-order fitting, third-order fitting, fourth-order fitting, fifth-order fitting, and sixth-order fitting are, respectively, performed on the errors between actual values and theoretical values of *l*_1_ during the movement of IN, with their fitting results shown as in Figure 8. The variance, standard deviation, and goodness of fit of each of the fitting values with the errors are shown in Table 4.

According to Figure 8 and Table 4, we choose third-order fitting as the optimal fitting curve of error compensation of *l*_1_ in IN direction as in the following equation:

(15) $$\begin{array}{c} \Delta l_{1}=-0.0027\beta^{3}+0.0526\beta^{2}-0.4178\beta -0.4263. \end{array}$$

#### 3.2.2. Error Calibration of *l*_1_ in EV Direction

The second-order fitting, third-order fitting, fourth-order fitting, fifth-order fitting, and sixth-order fitting are, respectively, performed on the errors between actual values and theoretical values of *l*_1_ during the movement of EV, with their fitting results shown as in Figure 9. The variance, standard deviation, and goodness of fit of each of the fitting values with the errors are shown as in Table 5.

According to Figure 9 and Table 5, we choose second-order fitting as the optimal fitting curve of error compensation of *l*_1_ in EV direction as in the following equation:

(16) $$\begin{array}{c} \Delta l_{1}=-0.0121\beta^{2}-0.2237\beta +0.2093. \end{array}$$

### 3.3. Calibration of *l*_2_ in IN/EV Direction

The result of *l*_2_ calibration in the direction of IN/EV is as in Figure 10, from which we can see that the error trends in IN/EV are also different, so we also calibrate them separately.

#### 3.3.1. Error Calibration of *l*_2_ in IN Direction

The second-order fitting, third-order fitting, fourth-order fitting, fifth-order fitting, and sixth-order fitting are, respectively, performed on the errors between actual values and theoretical values of *l*_2_ during the movement of IN, with their fitting results shown as in Figure 11. The variance, standard deviation, and goodness of fit of each of the fitting values with the errors are shown in Table 6.

According to Figure 11 and Table 6, we choose third-order fitting as the optimal fitting curve of error compensation of *l*_2_ in IN direction as in the following equation:

(17) $$\begin{array}{c} \Delta l_{2}=0.0027\beta^{3}-0.0591\beta^{2}+0.4172\beta +0.4266. \end{array}$$

#### 3.3.2. Error Calibration of *l*_2_ in EV Direction

The second-order fitting, third-order fitting, fourth-order fitting, fifth-order fitting, and sixth-order fitting are, respectively, performed on the errors between actual values and theoretical values of *l*_2_ during the movement of EV, with their fitting results shown as in Figure 12. The variance, standard deviation, and goodness of fit of each of the fitting values with the errors are shown in Table 7.

According to Figure 12 and Table 7, we choose second-order fitting as the optimal fitting curve of error compensation of *l*_2_ in EV direction as in the following equation:

(18) $$\begin{array}{c} \Delta l_{2}=0.0052\beta^{2}+0.2219\beta -0.2119. \end{array}$$

### 3.4. Calibration Results of *l*_1_ and *l*_2_

Through the above analysis, we can obtain the calibration results of the controlled lengths of *l*_1_ and *l*_2_ for the two linear actuators, which are the calibrated inverse solutions of positions.

#### 3.4.1. Lengths of *l*_1_ and *l*_2_ during DO (*α* > 0) Are as in (19)

(19) $$\begin{array}{c} l_{1}=l_{2}=\left|\left[\begin{array}{c} -55\\ 110c\alpha +4.5s\alpha -80\\ 110s\alpha -4.5c\alpha +406 \end{array}\right]\right|+\Delta l_{1}=\left|\left[\begin{array}{c} -55\\ 110c\alpha +4.5s\alpha -80\\ 110s\alpha -4.5c\alpha +406 \end{array}\right]\right|+1.4469\times 10^{-4}\alpha^{5}-0.0056\alpha^{4}+0.0781\alpha^{3}-0.4739\alpha^{2}+1.2322\alpha -0.136. \end{array}$$

#### 3.4.2. Lengths of *l*_1_ and *l*_2_ during PL (*α* < 0) Are as in (20)

(20) $$\begin{array}{c} l_{1}=l_{2}=\left|\left[\begin{array}{c} -55\\ 110c\alpha +4.5s\alpha -80\\ 110s\alpha -4.5c\alpha +406 \end{array}\right]\right|+\Delta l_{1}=\left|\left[\begin{array}{c} -55\\ 110c\alpha +4.5s\alpha -80\\ 110s\alpha -4.5c\alpha +406 \end{array}\right]\right|-0.0035\alpha^{2}+0.0106\alpha -1.1415. \end{array}$$

#### 3.4.3. Lengths of *l*_1_ and *l*_2_ during IN (*β* > 0) Are as in (21)

(21) $$\begin{array}{c} \left\{\begin{array}{c} l_{1}=\left|\left[\begin{array}{c} 120c\beta -4.5s\beta -175\\ 30\\ -120s\beta -4.5c\beta +406 \end{array}\right]\right|+\Delta l_{1}=\left|\left[\begin{array}{c} 120c\beta -4.5s\beta -175\\ 30\\ -120s\beta -4.5c\beta +406 \end{array}\right]\right|-0.0027\beta^{3}+0.0526\beta^{2}-0.4178\beta -0.4263,\\ l_{2}=\left|\left[\begin{array}{c} -120c\beta -4.5s\beta +175\\ 30\\ 120s\beta -4.5c\beta +406 \end{array}\right]\right|+\Delta l_{2}=\left|\left[\begin{array}{c} -120c\beta -4.5s\beta +175\\ 30\\ 120s\beta -4.5c\beta +406 \end{array}\right]\right|+0.0027\beta^{3}-0.0591\beta^{2}+0.4172\beta +0.4266. \end{array}\right. \end{array}$$

#### 3.4.4. Lengths of *l*_1_ and *l*_2_ during EV (*β* < 0) Are as in (22)

(22) $$\begin{array}{c} \left\{\begin{array}{c} l_{1}=\left|\left[\begin{array}{c} 120c\beta -4.5s\beta -175\\ 30\\ -120s\beta -4.5c\beta +406 \end{array}\right]\right|+\Delta l_{1}=\left|\left[\begin{array}{c} 120c\beta -4.5s\beta -175\\ 30\\ -120s\beta -4.5c\beta +406 \end{array}\right]\right|-0.0121\beta^{2}-0.2237\beta +0.2093,\\ l_{2}=\left|\left[\begin{array}{c} -120c\beta -4.5s\beta +175\\ 30\\ 120s\beta -4.5c\beta +406 \end{array}\right]\right|+\Delta l_{2}=\left|\left[\begin{array}{c} -120c\beta -4.5s\beta +175\\ 30\\ 120s\beta -4.5c\beta +406 \end{array}\right]\right|+0.0052\beta^{2}+0.2219\beta -0.2119. \end{array}\right. \end{array}$$

## 4. Experiments and Validation

In order to better verify the calibration effect of the PARR, we conducted relevant experiments in the directions of DO/PL and IN/EV, respectively. The method is to control the input of *l*_1_ and *l*_2_ and record the output angles of *α* and *β*, used to deduce the controlled lengths of *l*_1_ and *l*_2_ according to the calibration results. By comparing the inputs of *l*_1_ and *l*_2_ with the deduced lengths of *l*_1_ and *l*_2_ according to the calibration results, we can judge whether the calibration result is valid or not.

Firstly, we control the lengths of *l*_1_ and *l*_2_ using position controller for the two linear actuators to realize the movements of DO/PL and IN/EV, respectively. The lengths of *l*_1_ and *l*_2_ are controlled to run 1.875 mm (100 pulses) at a time. Then, we record the corresponding *α*, *β*, respectively. Lastly, the theoretical inputs of *l*_1_ and *l*_2_ are deduced based on the calibration results from (19) to (22) and the obtained *α*, *β*. By comparison with the theoretical inputs of *l*_1_ and *l*_2_ deduced from the inverse solution of positions without calibration, we can verify the effectiveness of the kinematic calibration of the parallel rehabilitation mechanism. The prototype of the 2-UPS/RRR PARR system used is as in Figure 13, with its human machine interface of the upper computer developed using C# programming language.

### 4.1. Results of DO

The experiment results of Δ*l*_1_ and Δ*l*_2_ in DO (Δ*l*_1_=Δ*l*_2_, *α* > 0) are as in Table 8, where Δ*l*_1ref_ denotes the controlled input length of *l*_1_ with its unit being mm, *α*_output_ is the detected angle of DO with its unit being ((°), *l*_1no_ represents the theoretical input of *l*_1_ without kinematic calibration, and *l*_1yes_ denotes the theoretical input of *l*_1_ with kinematic calibration, while err_no_ and err_yes_ represent the corresponding errors, respectively. For the reason that Δ*l*_1_=Δ*l*_2_, we just show *l*_1_ in Table 8 for the sake of simplification.

In order to show the error changes before and after calibration more intuitively during the DO movement, we compare the errors before and after calibration in the same figure, as in Figure 14.

### 4.2. Results of PL, IN, and EV

Similarly, we can obtain the experiment results of Δ*l*_1_ and Δ*l*_2_ in PL (Δ*l*_1_=Δ*l*_2_, *α* < 0), IN (*β* > 0), and EV (*β* > 0), with their errors before and after calibration shown as in Figures 15–17, respectively.

### 4.3. Discussion

#### 4.3.1. Comparison of Errors before and after Calibration

Based on the experiment results, the average errors before and after calibration are shown in Figure 18, where Err_*l*_1_uncali, Err_*l*_1_cali, Err_*l*_2_uncali, and Err_*l*_2_cali denote the errors of *l*_1_ without calibration, errors of *l*_1_ with calibration, errors of *l*_2_ without calibration, and errors of *l*_2_ with calibration, respectively. The average errors of *l*_1_ after calibration in the four directions have reduced by 98.32%, while the average errors of *l*_2_ after calibration in the four directions have reduced by 98.33%.

#### 4.3.2. Analysis of the Calibration Results

From (15) to (18), we can see that the calibration results of *l*_1_ and *l*_2_ in the IN and EV directions have almost the same behaviour and fitting orders, while from (13) and (14), we can see that *l*_1_ and *l*_2_ in the DO and PL directions have different behaviour and different fitting orders. The reason for this is that the two linear motors (SKF CAHB-10) used for actuating the two UPS kinematic branches are not servo motors and suffer from their nonlinear control, except for the mechanism's machining and assembly errors. In spite of this, we can see from Figure 18 that the errors after calibration become very small and the precision is significantly improved. The fact that that there is no need to calibrate the PARR before each use needs to be specially noted. The calibration results have been added in the control system to improve the control precision for isokinetic muscle strength exercise.

## 5. Conclusion

Kinematic calibration of the two UPS kinematic branches of the developed 2-UPS/RRR PARR is conducted and described in this paper in detail in order to improve the control precision for the rehabilitation training like isokinetic muscle strength exercise. Motion of each branch in different directions is fitted in high-order form according to experimental data. Variance, standard deviation, and goodness of fit are taken into consideration when choosing the best fitting curve. Experiments have been conducted, which show that the accuracy after calibration has been significantly improved and verify the effectiveness of the kinematic calibration.

In the future, we will study the repeatability performance of the kinematic calibration, as the repeatability of the kinematic calibration is an important aspect for the validation of the procedure. In addition, we will also focus on the kinematic calibration in the direction of AD/AB, compliant and interactive control strategies, as well as multimode rehabilitation training method.

## Figures and Tables

**Figure 1:** Structure of the ankle complex with its movement.

**Figure 2:** Mechanical structure of the developed 2-UPS/RRR PARR.

**Figure 3:** Coordinate system of the parallel mechanism and its UPS branch. (a) Schematic diagram of the mechanism. (b) UPS branch.

**Figure 4:** Error of *l*_1_ and *l*_2_ during calibration of DO/PL.

**Figure 5:** Error fitting of *l*_1_ and *l*_2_ during DO.

**Figure 6:** Error fitting of *l*_1_ and *l*_2_ during PL.

**Figure 7:** Error of *l*_1_ during calibration of IN/EV.

**Figure 8:** Error fitting of *l*_1_ during IN.

**Figure 9:** Error fitting of *l*_1_ during EV.

**Figure 10:** The error of *l*_2_ during calibration of IN/EV.

**Figure 11:** Error fitting of *l*_2_ during IN.

**Figure 12:** Error fitting of *l*_2_ during EV.

**Figure 13:** Prototype of the 2-UPS/RRR PARR.

**Figure 14:** Error comparison of *l*_1_ and *l*_2_ during DO.

**Figure 15:** Error comparison of *l*_1_ and *l*_2_ during PL.

**Figure 16:** Error comparison of *l*_1_ and *l*_2_ during IN.

**Figure 17:** Error comparison of *l*_1_ and *l*_2_ during EV.

**Figure 18:** Average error comparison of *l*_1_ and *l*_2_ before and after calibration.

**Table 1:** ROM of the AJC [24] and MAW of the designed PARR.

Motion direction	ROM (*°*)	MAW (*°*)
Dorsiflexion	20.3∼29.8	30.0
Plantarflexion	37.6∼45.8	45.0
Inversion	14.5∼22.0	22.0
Eversion	10.0∼17.0	22.0
Abduction	15.4∼25.9	36.0
Adduction	22.0∼36.0	36.0

**Table 2:** Fitting results of *l*_1_ and *l*_2_ during DO.

	2nd-order	3rd-order	4th-order	5th-order	6th-order
Var	0.0317	0.0310	0.0305	0.0190	0.0104
Std	0.1779	0.1776	0.1746	0.1379	0.1019
*R* ^2^	0.4062	0.4186	0.4280	0.6435	0.8051

**Table 3:** Fitting results of *l*_1_ and *l*_2_ during PL.

	2nd-order	3rd-order	4th-order	5th-order	6th-order
Var	0.037a	0.0351	0.035	0.0329	0.0326
Std	0.1923	0.1874	0.1872	0.1813	0.1805
*R* ^2^	0.6600	0.6772	0.6778	0.6979	0.7005

**Table 4:** Fitting results *l*_1_ during IN.

	2nd-order	3rd-order	4th-order	5th-order	6th-order
Var	0.0484	0.036	0.035	0.0349	0.0347
Std	0.2201	0.1898	0.1870	0.1869	0.1862
*R* ^2^	0.8707	0.9038	0.9067	0.9067	0.9075

**Table 5:** Fitting results of *l*_1_ during EV.

	2nd-order	3rd-order	4th-order	5th-order	6th-order
Var	0.0351	0.0349	0.0336	0.0336	0.0317
Std	0.1875	0.1869	0.1834	0.1834	0.1781
*R* ^2^	0.6881	0.6901	0.7015	0.7016	0.7186

**Table 6:** Fitting results of *l*_2_ during IN.

	2nd-order	3rd-order	4th-order	5th-order	6th-order
Var	0.0483	0.036	0.036	0.035	0.0347
Std	0.2197	0.1898	0.1870	0.187	0.1862
*R* ^2^	0.5239	0.6446	0.6552	0.6552	0.6581

**Table 7:** Fitting results of *l*_2_ during EV.

	2nd-order	3rd-order	4th-order	5th-order	6th-order
Var	0.0352	0.0349	0.0336	0.0336	0.0317
Std	0.1875	0.1869	0.1834	0.1834	0.1781
*R* ^2^	0.9098	0.9104	0.9137	0.9138	0.9187

**Table 8:** Experiment results of Δ*l*_1_ and Δ*l*_2_ in DO (Δ*l*_1ref_=Δ*l*_2ref_).

Δ*l*_1ref_	*α*_output_	*l*_1no_	*l*_1yes_	err_no_	err_yes_
1.875	0.748	1.423	1.974	0.452	−0.099
3.75	1.43	2.719	3.582	1.031	0.168
5.625	2.453	4.662	5.66	0.963	−0.035
7.5	3.427	6.51	7.471	0.99	0.029
9.375	4.498	8.54	9.44	0.835	−0.065
11.25	5.521	10.474	11.378	0.776	−0.128
13.125	6.495	12.312	13.293	0.813	−0.168
15	7.176	13.596	14.663	1.404	0.337
16.875	8.248	15.61	16.826	1.265	0.049
18.75	9.271	17.526	18.855	1.224	−0.105
20.625	10.293	19.436	20.803	1.189	−0.178
22.5	11.365	21.43	22.742	1.07	−0.242
24.375	12.387	23.326	24.532	1.049	−0.157
26.25	13.41	25.214	26.371	1.036	−0.121
28.125	14.481	27.183	28.56	0.942	−0.435

## Data Availability

All the data used to support the findings of this study are available from the corresponding author upon request.
